The article "Impact of Environmental Fluctuations on Stock Markets: Empirical Evidence from South Asia" was published in 2022. Journal: J Environ Public Health.

# Impact of Environmental Fluctuations on Stock Markets: Empirical Evidence from South Asia

**DOI:** 10.1155/2022/7692086

**Published:** 2022-07-14

**Authors:** R. M. Ammar Zahid, Muzammil Khurshid, Minha Waheed, Tajudeen Sanni

**Affiliations:** ^1^School of Accounting, Yunnan Technology and Business University, Kunming, China; ^2^Department of Banking and Finance, University of the Punjab, Gujranwala Campus, Gujranwala, Pakistan; ^3^Kampala International University, Kampala, Uganda

## Abstract

The proportionate use of energy represents economic activity as well as environmental degradation. This study intends to examine the volatility spillover of environmental fluctuations (energy prices) to the stock markets of south Asian countries (i.e., Bangladesh, India, and Pakistan). In this regard, the data have been gathered from the Thomson Reuters DataStream from 2013 to 2021. This study has applied the Granger causality test and ARCH-GARCH (1, 1). It concludes that the bidirectional causality exists between the environmental prices (i.e., energy market) and Bangladesh, Pakistan, and India stock markets (BSE-100, DSE-30, and KSE-100, respectively). The empirical findings of this study show that there are volatility spillovers from the energy to the stock markets of Pakistan and India. On the other hand, no volatility spillover is observed from the energy to the stock market of Bangladesh. Moreover, the study implies that investors should invest in these stock markets to reduce the risk involved with diversification.

## 1. Introduction

The environment is remarkably considered an essential part of accomplishing a country's economic goals. In the present decade, oil has become the basic necessity to run the economic activities of the countries, especially to stable the economy of the country [1, 2]. The recent demand for oil is 9%, reaching up to 17% in 2040 [3]. Several energy sources are being used, but oil consumption has reached one-third of overall energy consumption [4,5]. Furthermore, Aizenman and Pinto [6] have declared a relationship between the economic crisis and the volatility. This relationship is because the basic phenomenon behind both these factors is identical.

Over the decades, oil has held a pivotal role in environmental fluctuations and economic growth. Especially for oil-importing countries like India, Pakistan, and Bangladesh because the economies of these countries are highly dependent on oil. The dramatic increase in oil prices during the current decade has severely damaged the stock markets of India, Pakistan, and Bangladesh. According to the C.I.A. World Fact Book [7], India was declared the third-largest oil importer, while Pakistan was the thirty-fourth. Moreover, India consumes 4.521 million barrels per day, while Pakistan consumes 557,000 barrels per day. This research investigates the volatility spillovers from the energy market to the stock markets of some selected member countries of South Asia, namely, India, Pakistan, and Bangladesh. The study's research question is to what extent do the volatility spillovers from the oil market to selected south Asia member countries? The reason behind choosing these three countries relies on the fact that these countries import oil in a large quantity in this region. India, Pakistan, and Bangladesh are among the list of developing countries, and they use more oil to maintain their level of growth.

The article "Impact of Environmental Fluctuations on Stock Markets: Empirical Evidence from South Asia" was published in 2022. Journal: J Environ Public Health.

A growing body of literature has discussed the volatility spillover from energy consumption to stock markets in developed and developing countries [8–14]. The primary study in this regard was stepped by Hamilton [15] by focused on the impact of oil prices on the economy of the U.S. and found that sharp fluctuation in oil prices has a significant impact on the economy. Moreover, Basher and Sadorsky [16] identified the role of oil prices on 21 emerging stock markets by applying a multifactor model and found the significant impact of oil prices on these emerging markets. Khalfaoui, Boutahar, and Boubaker [8] have studied the oil volatility spillovers and G7 stock markets by employing multivariate wavelet and GARCH models. The analysis results provide considerable evidence of volatility spillovers from the oil market to the stock markets of G7 countries.

After examining all these studies, a mixed conclusion can be drawn because some studies suggest that the volatility is transmitted from the oil market to the stock markets of different countries; on the other hand, some studies prove that there is no transmittal of volatility from the market of oil to the stock of different countries. The findings vary from country to country and analyzed periods [17–21]. This difference in findings may be due to the methodology, model, time, or data set. This study is an effort to fill the gap in the literature on the subject of volatility transmission from the environmental fluctuations to the stock markets of south Asian countries by using the ARCH–GARCH model to observe the transmittal of instability from oil to the stock markets of south Asian countries, namely, Pakistan, India, and Bangladesh.

Moreover, our study results exhibit significant energy fluctuation spillovers to the stock exchanges of India and Pakistan. Still, there are no volatility spillovers from the oil market to the stock market of Bangladesh. Moreover, the study suggests that there is a need that economists, investors, and policymakers should keep an eye on the international oil market to avoid the risk. Furthermore, the results of this study are fruitful for traders, portfolio makers, policymakers, and investors interested in these emerging markets.

The article "Impact of Environmental Fluctuations on Stock Markets: Empirical Evidence from South Asia" was published in 2022. Journal: J Environ Public Health.

## 2. Materials and Methods

The data of this study contains daily closing prices of oil West Texas Intermediate (WTI) and stock market indices of selected South Asian countries: Pakistan, India, and Bangladesh. The benchmark indices of Pakistan, India, and Bangladesh stock markets have been utilized in this study since only these three countries in the region have well-developed stock markets and indices data. The benchmark index of the Pakistan Stock Exchange is KSE-100 (Karachi Stock Exchange); for Bangladesh Stock Exchange, it is DSE-30 (Dhaka Stock Exchange); and for the Indian Stock Exchange, it is BSE-100 (Bombay Stock Exchange). Daily stock and oil prices from Jan 30, 2013, to Jun 14, 2021, have been taken to make a better empirical analysis. The daily data was gathered from the Thomson Reuters data stream for analysis. Moreover, the days on which holidays are observed in the stock and oil markets have been excluded from the data stream. The second filtration is that the data of stock and oil prices have been provided in the U.S. dollar.

In this study, the unit root test has been conducted, i.e., the augmented Dickey–Fuller Test (ADF) and the Philips–Perron test (PP), to test whether the time series data is stationary or not nonstationary. The null hypothesis (H0) for ADF Test and PP Test is that there is a unit root in the series or the data is not stationary, while the H_1_ demonstrates that the time series data is stationary or there is no unit root in the data. This study applies granger causality and the ARCH-GARCH (1, 1) model to examine the spillover of volatility from oil to the stock markets, namely, the Karachi Stock Exchange, Bombay Stock Exchange, and Dhaka Stock Exchange. GARCH (1.1) represents one ARCH term and one GARCH term. There are two conditions to apply this model, i.e.,

- There should be clustering volatility
- There should be an ARCH effect

Here clustering volatility demonstrates that the period of high volatility should be followed by the period of high volatility. The period of low volatility should be followed by a period of low volatility for a long period. The GARCH (1, 1) model determines transmission from the oil market to Pakistan, Bangladesh, and the Indian stock market. There are two equations in this model first one is the mean equation, and the second one is the variance equation. The mean equation for this model is as follows:

(1) $$\begin{array}{c} R{}_{t}=\mu +\rho R_{t-1}+\varepsilon {}_{t}, \end{array}$$

where *R*_t_ represents the return series from the oil or stock market and *ε*_*t*_ represents the residual series that are normally distributed, having a mean of zero. Now moving toward the conditional variance equation of this model, it is given as follows:

(2) $$\begin{array}{c} H{}_{t}=\omega +\alpha \varepsilon_{t-1}^{2}+\beta h_{t-1}. \end{array}$$

Note that *H*_*t*_ is the representation of the conditional variance that depends on the level of mean volatility (*ω*), *ε*^2^_*t*−1_ represents the effect of news from the previous period, whereas *h*_*t*−1_ represents the conditional variance from the previous period. The sum of *α* and *β* is measured by how long volatility prevails derived from a shock.

The article "Impact of Environmental Fluctuations on Stock Markets: Empirical Evidence from South Asia" was published in 2022. Journal: J Environ Public Health.

## 3. Results and Discussion

Table 1 demonstrates the findings of descriptive statistics for stock markets and oil market returns from Jan 30, 2013, to Jun 14, 2021. It represents that the average daily return earned by the oil market is 0.0003 having a standard deviation of 0.034, which is higher in comparison to the stock markets. This shows that the return of the oil market is more volatile compared to the stock markets and the reason behind this is that crude oil is well known and significant in the international market. The standard deviation of Karachi stock returns came out to 0.014, which suggests that the returns of Karachi stocks are less volatile in comparison to the oil market and more volatile in comparison to the returns of the Dhaka stock exchange. Talking about the Bombay stock exchange, the average daily return from 2013 to 2021 is observed to be 0.0007, which is low compared to the Karachi stock exchange and high in comparison to both Dhaka stock exchanges and the crude oil market.

Table 2 shows the results of the augmented Dickey–Fuller Test with the trend and without trend. The purpose of this test is to know about the stationary of the data. This test is applied to examine whether the data is stationary or not. The critical values for without trend at 1%, 5%, and 10% are −2.580, −1.950, and −1.620, respectively, while for with trend it is −3.960, −3.410, and −3.120. The alternative hypothesis will be accepted, and the null hypothesis will be rejected if the test statistic value comes out to be greater than the critical value. Normally we compare test statistics with the 5% critical value. Acceptance of H_1_ represents the stationary of data. So from the results of the analysis, we can conclude that our data for stock markets and the oil market is stationary. We do not need to make a difference to make the data stationary. On the whole, results came out that the H_1_ is accepted and the H_0_ is rejected.

The article "Impact of Environmental Fluctuations on Stock Markets: Empirical Evidence from South Asia" was published in 2022. Journal: J Environ Public Health.

Table 2 represents the analysis done for the ADF and Phillips–Perron test with the trend and without trend to check the stationary of stock and crude oil market. The critical values for without trend at 1%, 5%, and 10% is −2.580, −1.950, and −1.620, respectively, while for with trend it is −3.960, −3.410, and −3.120. The alternative hypothesis will be accepted, and the null hypothesis will be rejected if the test statistic value is higher than the critical value.

As the test statistics value is higher than the critical value, it can be evaluated that the data is stationary. This demonstrates that the H_0_ is rejected and the H_1_ is accepted. The next step is to implement the GARCH (1, 1) model, and before running this model, it will be checked whether there is clustering volatility or not and whether the data has an arch effect or not. The GARCH model will only be implemented if there is clustering volatility and also if there is a representation of the ARCH effect in the data.

Figure 1 represents the clustering volatility of the residuals, and it can be evaluated from the graph that there is clustering volatility in the data as the period of low volatility is followed by low volatility, and the period of high volatility is followed by a period of high volatility for a prolonged period. This fulfills the one condition to implement the GARCH (1, 1) model. Now we need to check the second condition that whether there is the representation of an ARCH effect in the data or not, and this can be done through the LM test. If the value of probability came out greater than 5 in the LM test, then there will be no ARCG effect, and if the probability is less than 5, there will be an ARCH effect in the data.

Table 3 indicates the Granger causality test for energy and the stock market. The results demonstrate bidirectional causality between the WTI oil market and Bangladesh, Pakistan, and India. These results are similar to Ho and Huang [22] because they also found causality between oil and the Indian stock market. Moreover, bidirectional causality runs between the Bombay stock market and the Bangladeshi stock market. The noteworthy point is that there is no causality between the stock market of Bangladesh and Pakistan.

Table 4 represents the LM test to verify the condition of the Arch effect, and it represents that the condition of the ARCH effect is fulfilled as it can be seen that the probability is less than 5, so we can accept H1 and reject H0, which is the demonstration of an ARCH effect in the data. Now, on the whole, we can say that the GARCH (1, 1) model can be implemented as there is clustering volatility along with the ARCH effect in the data.

The article "Impact of Environmental Fluctuations on Stock Markets: Empirical Evidence from South Asia" was published in 2022. Journal: J Environ Public Health.

Table 5 represents the transmittal of volatility from the oil market to the stock markets of India, Pakistan, and Bangladesh using the GARCH (1, 1) model. However, the results from the GARCH model came out that there is transmittal of volatility from the oil market to the stock markets of India and Pakistan, and the results for the Bangladesh stock market are not significant means there is no spillover effect in that market. These results are evaluated from the *P* > |z| value. If the *P* > |z| value came out to be less than 5%, then there is volatility spillover, and the results are significant. On the other hand, if the *P* > |z| value came out to be greater than 5%, the results are insignificant, and there is no spillover effect. As the results of this study came out to be smaller than 5%, that is , 0.00 for Pakistan and the Indian stock market, this means that volatility will be transmitted from the oil market to the stock markets of Pakistan and India. On the other hand, the results for the Bangladesh stock market do not come out to be significant as the *P* >|z| value is greater than 5%, that is, 0.160 in the Bangladesh stock market. From these results, it can be originated that if any disturbance came in the oil market, then that disturbance will also affect the stock markets of Pakistan and India. At the same time, there will be no effect on the stock market of Bangladesh.

## 4. Conclusions

This paper aims to determine whether there are environmental fluctuations spillover from the energy to stock markets of south Asian countries (Pakistan, India, and Bangladesh). For this purpose, the ARCH-GARCH model and granger causality tests have been applied. The sample era of this study is from the year 2013 to 2021. This study employs the date of daily closing prices for stock prices and crude oil prices from the period starting from Jan 30, 2013, to Jun 4, 2021. The empirical findings of this study indicate that the Karachi stock exchange and Bombay stock exchange are influenced by the oil market, while the results for the Dhaka stock exchange are not the same.

The study concludes that bidirectional causality exists between the WTI oil market and Bangladesh, Pakistan, and India. Moreover, the findings represent that there is no influence of the oil market on the stock market of Dhaka. This means that the result of the study indicates a transmittal of volatility from the oil market to the stock markets of Pakistan and India. Still, there are no spillover effects from the oil market to the Bangladesh stock market. It can be concluded from these results that the reason for this transmittal from the oil market to the stock markets of Pakistan and India may be that these countries import a large amount of oil to fulfill the need of their people. Malik [23] has found that mostly the countries which import oil are affected due to any fluctuation that comes in the crude oil market. Similarly, the stock markets of these oil-importing countries are also affected by crude oil prices because any fluctuation directly influences earnings along with the cash flow streams in the prices of crude oil. This has been discussed above that when the prices of oil increase in the international oil market, the production and input costs increase, reducing the earnings of an organization and the share prices go down. The further reduction in the prices of shares leads to reducing the dividends and profits of an organization, which reduces domestic and foreign investment.

The article "Impact of Environmental Fluctuations on Stock Markets: Empirical Evidence from South Asia" was published in 2022. Journal: J Environ Public Health.

On the other hand, when oil prices decrease, input and production cost decreases, and earnings and investment increase. So, the transmittal of instability from the oil market to the stock markets of Pakistan and India can be observed in this study. At the same time, Bangladesh's results are not significant, meaning there are no spillover effects in the stock market in Bangladesh. The information provided in this paper will provide a ground for policymakers and investors to take more effective and profitable decisions.

This study suggests that there is a need that economists, investors, and policymakers to keep an eye on the information that comes from the international oil market. On the grounds of the results, this study recommends that to balance their budget India and Pakistan should make an effort to balance their import and exports as they cannot reduce their consumption of oil due to the lack of alternatives. As the level of oil consumption is increasing day by day in Pakistan, India, and Bangladesh, the Government of these countries needs to facilitate the transporters for the consumption of fuel. As debated above, a group of studies has investigated the transmission of volatility from the market of oil to the stock markets. Still, a very limited number of studies have observed the spillover effect from the oil market to the stock markets of Pakistan, India, and Bangladesh using the GARCH (1, 1) model.

This study has considered only three countries of South Asia, but in the future study can be done on all the countries of South Asia. Other regions like European Union can also be examined. Similarly, a comparison of volatility spillover can also be done between developed and developing countries. As among all other models, I have used the ARCH-GARCH model for my study in the future; any other methodology like ARMA (1, 1) or any other can be used to observe the transmittal of volatility from the oil market to Pakistan, Bangladesh, and Indian stock markets.

The article "Impact of Environmental Fluctuations on Stock Markets: Empirical Evidence from South Asia" was published in 2022. Journal: J Environ Public Health.

## Figures and Tables

**Figure 1:** Clustering volatility of the residuals.

**Table 1:** Descriptive statistics.

Variables	DSE	KSE	BSE	Oil
Mean	0.0003	0.00082	0.0007	0.0003
S.D	0.011	0.0148	0.013	0.034
Kurtosis	16.460	59.54	37.15	133.80
Skewness	0.190	2.680	1.593	5.128
Maximum	0.102	0.249	0.190	0.710
Minimum	−0.086	−0.097	−0.082	−0.323
Observations	1453	1453	1453	1453

**Table 2:** Results of unit root test.

	With trends		Without trends	
Country	ADF	PP test	ADF	PP test
Bangladesh	−45.834	−44.974	−45.415	−44.377
Pakistan	−51.015	−48.941	−50.630	−48.386
India	−46.754	−45.846	−46.610	−45.583
Oil	−50.529	−51.448	−50.496	−51.365

**Table 3:** Summary statistics for granger causality test.

Null hypothesis	*χ*2	Lag	*p* value	Null Hypothesis	*χ*2	Lag	*p* value
B.D. ≠> IND	0.21^*∗∗*^	1	0.02	PAK ≠> BD	0.43	1	0.23
BD ≠> PAK	0.41	1	0.41	PAK ≠> IND	0.45^*∗∗*^	1	0.01
BD ≠> oil	0.24^*∗∗∗*^	1	0.001	PAK ≠> oil	1.65^*∗∗∗*^	1	0.001
IND ≠> BD	1.24^*∗∗*^	1	0.01	Oil ≠> BD	3.45^*∗∗*^	1	0.04
IND ≠> PAK	0.43	1	0.21	Oil ≠> IND	0.90^*∗∗∗*^	1	0.001
IND ≠> oil	1.45^*∗∗∗*^	1	0.001	Oil ≠> PAK	3.54^*∗∗∗*^	1	0.001

Notes: “≠>” means “does not Granger-cause.” the Schwarz information criterion (SIC) is used. ^*∗∗∗*^, ^*∗∗*^, and ^*∗*^ to indicate a rejection of the null hypothesis.

**Table 4:** LM test for ARCH effect.

Lags(*p*)	chi2	Df	Prob > chi2
1	24.672	1	0.0000

**Table 5:** ARCH family regression.

Sample: 30 Jan 13 to 14 Jun 21 but with gaps			No. of observations = 1453			
Distribution: Gaussian			Prob > chi2 = 0.0000			
OIL WTI	Coef.	Std. Err.	*Z*	P>|z|	[95% conf. Interval]	
OILWTI	—					
DSE-30	0.062	0.044	1.41	0.160	0.0245	0.1491
KSE-100	0.359	0.042	8.41	0.000	0.2759	0.4438
BSE-100	0.654	0.051	12.72	0.000	0.5533	0.7549
-cons	−0.0004	0.0005	−0.68	0.495	−0.0015	0.0007
ARCH	0.8013	0.046	17.42	0.000	0.711	0.891
L1.						
GARCH						
L1.	0.1056	0.0324	3.26	0.001	0.0421	0.169
−cons	0.0002	0.00002	9.21	0.000	0.0002	0.0003

## Data Availability

The datasets used and analyzed during the current study are available from the Thomson Rutters eikon DataStream.
